# A Network Pharmacology Method Combined with Molecular Docking Verification to Explore the Therapeutic Mechanisms Underlying Simiao Pill Herbal Medicine against Hyperuricemia

This article has been retracted.

**DOI:** 10.1155/2023/2507683

**Published:** 2023-02-09

**Authors:** Yue Qian, Jiazhen Yin, Juemin Ni, Xiaona Chen, Yan Shen

**Affiliations:** ^1^Rehabilitation Center, Hangzhou Wuyunshan Hospital (Hangzhou Institute of Health Promotion), Hangzhou 310000, China; ^2^Department of Nephrology, Hangzhou TCM Hospital of Zhejiang Chinese Medical University (Hangzhou Hospital of Traditional Chinese Medicine), Hangzhou 310000, China; ^3^Department of Nursing, Hangzhou Wuyunshan Hospital (Hangzhou Institute of Health Promotion), Hangzhou 310000, China

## Abstract

**Objective:**

Hyperuricemia (HUA) is a common metabolic disease caused by disordered purine metabolism. We aim to reveal the mechanisms underlying the anti-HUA function of Simiao pill and provide therapeutic targets.

**Methods:**

Simiao pill-related targets were obtained using Herbal Ingredients' Targets (HIT), Traditional Chinese Medicine Systems Pharmacology (TCMSP), and Traditional Chinese Medicine Integrated Database (TCMID). HUA-associated targets were retrieved from GeneCards, DisGeNET, and Therapeutic Targets Database (TTD). Protein-protein interaction (PPI) network was constructed using the Search Tool for the Retrieval of Interacting Genes/Proteins (STRING) database, ggraph and igraph R packages. Gene Ontology (GO) and Kyoto Encyclopedia of Genes and Genomes (KEGG) analyses were performed using ClusterProfiler. The top 10 core targets were identified through cytoHubba. Molecular docking was conducted using PyMOL and AutoDock high-performance liquid chromatograph (HPLC) analysis was performed to identify effective compounds of Simiao pill.

**Results:**

Simiao pill-HUA target network contained 80 targets. The key targets were mainly involved in inflammatory responses. Insulin (INS), tumor necrosis factor (TNF), interleukin-6 (IL6), interleukin 1 beta (IL1B), vascular endothelial growth factor A (VEGFA), leptin (LEP), signal transducer and activator of transcription 3 (STAT3), C-C motif chemokine ligand 2 (CCL2), interleukin-10 (IL10), and toll like receptor 4 (TLR4) were the top 10 targets in the PPI network. GO analysis demonstrated the main implication of the targets in molecular responses, production, and metabolism. KEGG analysis revealed that Simiao pill might mitigate HUA through advanced glycation end-product- (AGE-) receptor for AGE- (RAGE-) and hypoxia-inducible factor-1- (HIF-1-) associated pathways. IL1B, IL6, IL10, TLR4, and TNF were finally determined as the promising targets of Simiao pill treating HUA. Through molecular docking and HPLC analysis, luteolin, quercetin, rutaecarpine, baicalin, and atractylenolide I were the main active compounds.

**Conclusions:**

Simiao pill can mitigate HUA by restraining inflammation, mediating AGE-RAGE- and HIF-1-related pathways, and targeting IL1B, IL6, IL10, TLR4, and TNF.

## 1. Introduction

Hyperuricemia (HUA) is a common metabolic disorder triggered by abnormal purine metabolism, with a rising incidence worldwide [1, 2]. It has been reported that the prevalence of HUA was 11.9–25.0% in Europe, 11.3–47% in the United States, 26.8% in Japan, and 13.1–13.3% in China [3]. The onset of HUA is dominantly due to the boosted formation or decreased excretion of uric acid [4]. Uric acid is the product of purine breakdown, which circulates in the ionized form of urate at the normal physiological pH of 7.4. Purine metabolism primarily occurs in the liver, also produced in any other tissue with xanthine oxidase (intestines) [5]. HUA can lead to gout and kidney stones [6, 7], and it is closely linked with the development of cardiovascular disease [8]. Although the exact cause and pathogenesis remain unclear, inflammation and oxidative stress have been demonstrated to be closely associated with the pathological mechanisms of HUA [9]. Noteworthily, HUA tends to be asymptomatic, bringing a challenge to the management and treatment of HUA.

In the last decades, the therapeutic strategies of HUA have counted on the decline in uric acid. Xanthine oxidase inhibitors such as allopurinol [10] and febuxostat [11] have been regarded as promising uric acid-lowering drugs to treat HUA [12]. Despite significant improvements in anti-HUA agents, current drug therapy is insufficient to cure HUA and prevent the onset of HUA-associated disorders. Therefore, safer and more effective drugs for treating HUA are desperately needed.

Traditional Chinese medicine (TCM) has gained global attention owing to its favorable efficacy and safety in the treatment of various diseases, and the application of herbal remedies is increasing worldwide. Plants have been the main source of tradition medicines since ancient times [13]. Some Chinese herbs or their active ingredients, such as plantain [14] and berberine [15], have exhibited curative potential for HUA. Simiao pill, a TCM formula, consists of Rhizoma Atractylodis, Cortex Phellodendri, Radix Achyranthis Bidentatae, and Semen Coicis at the ratio of 1 : 2 : 1 : 2 [16, 17]. Pharmacological research has indicated that Simiao pill contains a variety of natural active compounds, such as flavonoids and phenols [18]. Interestingly, recent studies have demonstrated that some phytochemicals including flavonoids and phenols possess antioxidative activity, which benefit to the treatment of various diseases and health care [13, 19, 20]. Simiao pill is used as a damp-removing agent with the function of eliminating heat and dispelling dampness, which can treat damp-heat betting-induced arthralgia [21]. Modern pharmacological study has indicated that Simiao pill has multiple pharmacological properties, including anti-inflammation [22], and it has been utilized to treat rheumatoid arthritis [23]. Interestingly, recent research has indicated the anti-HUA effect of Simiao pill [24]. Nevertheless, research into the potential anti-HUA function and its mechanisms is still lacking.

Network pharmacology is an emerging tool for data collection and analysis of TCM, which combines bioinformatics with system medicine [25, 26]. In recent years, network pharmacology has been broadly used for investigation into TCM due to its capability of clarifying the features of multiple ingredients and targets of TCM [26]. Herein, we probed into the active components of Simiao pill and relevant therapeutic targets based on these facts. Through network pharmacology and molecular docking, we aim to uncover the mechanisms underlying Simiao pill treating HUA, thereby providing therapeutic targets against HUA. Besides, we conducted high-performance liquid chromatograph (HPLC) analysis for quality control and verification of the potential active ingredients of Simiao pill against HUA. The workflow of this study is shown in Figure 1.

## 2. Materials and Methods

### 2.1. Databases and Analysis Tools

Platforms or tools utilized in this study are shown as follows: Herbal Ingredients' Targets (HIT; v2.0; http://hit2.badd-cao.net), Traditional Chinese Medicine Systems Pharmacology (TCMSP; http://tcmspw.com/tcmsp.php), Traditional Chinese Medicine Integrated Database (TCMID; v2.0; http://www.megabionet.org/tcmid/), GeneCards (v3.0; https://www.genecards.org/), DisGeNET (v7.0; http://www.disgenet.org/), Therapeutic Targets Database (TTD; https://idrblab.org/ttd/), PubChem (https://pubchem.ncbi.nlm.nih.gov), UniProt (https://www.uniprot.org/), VennDiagram (v1.7.3; http://bioinfogp.cnb.csic.es/tools/venny/index.html), Cytoscape (v3.7.2, http://www.cytoscape.org/), Search Tool for the Retrieval of Interacting Genes/Proteins (STRING; https://string-db.org/cgi/input.pl), ggraph (v2.0.5), igraph (v1.3.1), cytoHubba (v0.1), Metascape (http://metascape.org/), ClusterProfiler (v4.0, https://bioconductor.org/packages/release/clusterProfiler.html), circlize R package (v0.4.15), Research Collaboratory for Structural Bioinformatics Protein Data Bank (RCSB PDB, https://www.rcsb.org/), PyMOL (v2.1), AutoDock (v1.5.6), ZINC (https://zinc.docking.org/), and Open Babel graphical user interface (GUI; v2.3.1).

### 2.2. Screening of Active Components of Simiao Pill and Relevant Targets

Active components of Simiao pill were retrieved from HIT [27], TCMSP [28], and TCMID [29] databases. After duplication deletion, the structures of active components were obtained from the PubChem database [30].

Absorption, distribution, metabolism, and excretion (ADME) filtration is of great significance to the development of drugs [31, 32]. Based on ADME properties, the criteria of “quantitative estimate of drug − likeness (QED) ≥ 0.2” [33] was applied to sort out active components of Simiao pill. Then, targets related to active components were obtained from the HIT database. Some target genes repeated were excluded. The targets were standardized using the UniProt database [34] with the species set to “*Homo sapiens*.”

### 2.3. Collection of HUA-Related Targets

Potential HUA-related targets were obtained from GeneCards [35], DisGeNET [36], and TTD [37] databases with the search term “hyperuricemia”. Similarly, HUA-associated targets repeated were eliminated. The obtained targets were standardized using the UniProt database with the species limited to “*Homo sapiens*.”

### 2.4. Identification of Simiao Pill-HUA Intersection Targets and Protein-Protein Interaction (PPI) Network Analysis

Common targets of Simiao pill and HUA were acquired using VennDiagram. Then, overlapping targets of active components of Simiao pill and HUA were entered into the STRING database [38] to establish the PPI network. The ggraph and igraph R packages were utilized to visualize the protein interactions. The nodes of the PPI network represent proteins, and the edges represent the relations between two proteins. In the current study, we set the species to “*Homo sapiens*” and the confidence score of “>0.4” to screen out candidate targets. The other parameters for PPI network were default: network type = full STRING network; size cutoff = no more than 10 interactors. Besides, the cytoHubba plugin was used for screening the core targets (top 10) with the parameters set to “ranking method = maximal clique centrality (MCC); Hubba nodes = top 10 nodes ranked by MCC (default)”.

### 2.5. Gene Ontology (GO) and Kyoto Encyclopedia of Genes and Genomes (KEGG) Pathway Enrichment Analyses

In this study, Metascape was applied for GO and KEGG pathway enrichment analyses with the species of “*Homo sapiens*.” Metascape is a web-based portal, which provides gene annotation and analysis resource [39]. GO analysis comprises biological process (BP), cellular component (CC), and molecular function (MF). We performed KEGG analysis to find out the pathway mechanisms of HUA associated with the overlapping targets. ClusterProfiler in R package [40] was utilized to visualize the results of GO and KEGG pathway enrichment. To determine whether the target gene set is significantly associated with specific gene ontology and pathways, the hypergeometric distribution model was used. The following hypergeometric distribution formula was applied:

(1) $$\begin{array}{c} P=1-\overset{k-1}{\underset{i=0}{\sum }}\frac{\left(\begin{array}{c} M\\ i \end{array}\right)\left(\begin{array}{c} N-M\\ n-i \end{array}\right)}{\left(\begin{array}{c} N\\ n \end{array}\right)}, \end{array}$$

where *N* is the total number of genes; *M* is the number of annotated genes in GO or KEGG pathways; *n* is the number of imported target genes; and *k* is the number of common genes. *P* value < 0.01 was considered statistically significant [41].

### 2.6. Screening of GO-KEGG-Based Hub Targets

Top 10 hub genes originating from GO functional annotation and KEGG pathway analyses were obtained using the cytoHubba plugin. Similarly, the following parameters of cytoHubba were applied: ranking method = maximal clique centrality (MCC); Hubba nodes = top 10 nodes ranked by MCC (default). The circlize R package was applied to visualize the hub target network.

### 2.7. Molecular Docking

Molecular docking was conducted to verify the interactions between active components and core target proteins of Simiao pill treating HUA. Crystal structures of candidate proteins were downloaded from RCSB PDB [42]. PyMOL and AutoDock tools were used to remove water molecules and ligands, add hydrogen, optimize amino acids, and calculate charges for the structures. The structures were saved in PDB format. Subsequently, 3D structures of the active components in mol2 format were downloaded from ZINC [43]. All structure files were converted into PDBQT format by Open Babel GUI software. Docking pairs simultaneously that met the criteria of the binding free energy < −5.0 kcal/mol and the formation of hydrogen bonds were considered effective [44] and used for subsequent analysis. Finally, AutoDock Vina was used for molecular docking, and PyMOL was for visualization of the results.

### 2.8. Preparation of Simiao Pill Sample Solutions and Standard Solutions

Simiao pill used in this study was provided by the Department of Pharmacy of Hangzhou Wuyunshan Hospital (Hangzhou, China). All the preparation procedures conformed to the standards of the Chinese Pharmacopoeia (2020 edition). Briefly, 0.2 g of Simiao pill powder was accurately weighed out and added into 40 mL solution of hydrochloric acid-methanol (1 : 100) for 45 min of ultrasound (power: 250 W; frequency: 33 kHz). After cooling, the hydrochloric acid-methanol solution (1 : 100) was added to 50 mL, followed by shaking and filtering. The subsequent filtrate was obtained and injected through a 0.22 *μ*m filter membrane for subsequent high-performance liquid chromatograph (HPLC) analysis.

Ingredients used to prepare the standard solutions were purchased from Shanghai Yuanye Bio-Technology Co., Ltd, and Shanghai Chunxiao Bio-Technology Co., Ltd (Shanghai, China). The ingredients used were as follows: chlorogenic acid (#B20782, HPLC ≥ 98%, Yuanye), magnoflorine (#B20882, HPLC ≥ 98%, Yuanye), berberine hydrochloride (#B21449, HPLC ≥ 98%, Yuanye), luteolin (#B20888, HPLC ≥ 98%, Yuanye), palmitic acid (#1957-10-3, HPLC ≥ 98%, Chunxiao), wogonin (#B20489, HPLC ≥ 98%, Yuanye), atractylenolide I (#B20054, HPLC ≥ 98%, Yuanye), osthole (#B21152, HPLC ≥ 98%, Yuanye), quercetin (#B20527, Yuanye), rutaecarpine (#B21314, HPLC ≥ 98%, Yuanye), paeonol (#B20266, HPLC ≥ 98%, Yuanye), kaempferol (#B21126, HPLC ≥ 98%, Yuanye), baicalin (#B20570, HPLC ≥ 98%, Yuanye), vitamin E (#B21296, HPLC ≥ 97%, Yuanye), and phytosterol (#B20272, HPLC ≥ 98%, Yuanye). For the preparation of standard solutions, 10 mg of these reference sample components was accurately weighed and dissolved in 10 mL methanol, respectively. Then, equal volumes (10 mL) of these stock solutions were blended to obtain the mixed standard solution.

### 2.9. HPLC Analysis

HPLC analysis was performed on the 1260 Infinity II liquid chromatograph system (Agilent, Palo Alto, California, USA) with 10 *μ*L mixed standard solution and sample solution, respectively, injected. The mobile phase consisted of acetonitrile (A) and 0.1% phosphoric acid (B). The procedure of gradient elution was set as follows: 0~30 min, 7%~18%A; 30~45 min, 18%~22.5%A; 45~50 min, 22.5%~24%A; 50~65 min, 24%~48%A; 65~75 min, 48%~51%A; 75~90 min, 51%~70%A; 90~95 min, 70%~7%A; and 95~100 min, 7%~7%A. The operation time was set to 100 min, the flow rate to 1 mL/min, the column temperature to 30°C, and the detection wavelength to 280 nm.

## 3. Results

### 3.1. Identification of Simiao Pill-HUA Candidate Targets

After retrieval from HIT, TCMSP, and TCMID databases, 282 active compounds of Simiao pill were obtained, excluding those repeated or without PubChem ID (Table S1). A total of 264 active compounds met the criterion of “QED ≥0.2” and were used for the following selection of candidate target genes (Table S2). Also, we acquired 606 target genes related to the active compounds of Simiao pill after searching from the HIT database (Table S3). Moreover, 303 HUA-associated target genes were obtained from GeneCards, DisGeNET, and TTD databases, excluding those repeated or without UniProt ID (Table S4). Significantly, we acquired the intersections between the above 606 active compound-related and 303 disease-related genes, resulting in 80 Simiao pill-HUA targets (Table 1 and Figure 2).

### 3.2. PPI Network of Simiao Pill-HUA Common Targets

To clarify the potential links among the identified 80 targets, the PPI network analysis was performed. In the current research, the PPI network included 79 nodes (proteins; degree ≥ 2) and 1,083 edges (interaction pairs; score > 0.4). The top 10 hub proteins (red nodes) were presented as follows: insulin (INS; degree = 66), tumor necrosis factor (TNF; degree = 61), interleukin-6 (IL6; degree = 60), interleukin 1 beta (IL1B; degree = 55), vascular endothelial growth factor A (VEGFA; degree = 51), leptin (LEP; degree = 50), signal transducer and activator of transcription 3 (STAT3; degree = 48), C-C motif chemokine ligand 2 (CCL2; degree = 46), interleukin-10 (IL10; degree = 46), and toll-like receptor 4 (TLR4; degree = 43) (Table S5 and Figure 3). These core genes might be significantly implicated in the pathogenesis of Simiao pill treating HUA.

### 3.3. GO and KEGG Pathway Enrichment Analyses

To explore the biological functions of 80 potential targets, GO enrichment analysis was conducted. In this study, 1,612 BP, 19 CC, and 50 MF terms correlated with the 80 targets were obtained (*P* value < 0.01) (Table S6). Then, the top 5 enriched GO items were, respectively, screened out of BP, CC, and MF terms. The results of GO analysis showed that the candidate targets were mainly concentrated in BPs, including response to peptide and regulation of small molecule metabolic process; CCs, such as membrane raft and membrane microdomain; MFs, such as signaling receptor activator activity and receptor ligand activity (Table 2 and Figure 4(a)). Also, we applied KEGG pathway analysis to probe into the pathway mechanisms underlying these targets. The top 15 enriched KEGG pathways were identified, including the AGE-RAGE signaling pathway in diabetic complications and HIF-1 signaling pathway (*P* value < 0.01) (Table 3 and Figure 4(b)).

### 3.4. Identification of Hub Genes Based on GO and KEGG Analyses

To find out which target acts as a vital switch in the regulation of the above 15 enriched biological functions and 15 pathways, we further screened out the hub targets using the cytoHubba plugin. The interaction network of the candidate targets; 15 GO terms of top 5 BP, CC, and MF; and top 15 KEGG pathways is shown in Figure 5(a). According to the maximal clique centrality (MCC) scores, the 10 hub GO-KEGG genes were acquired, namely, TNF (MCC score = 23), IL1B (MCC score = 20), IL6 (MCC score = 18), transforming growth factor beta 1 (TGFB1; MCC score = 17), interferon gamma (IFNG; MCC score = 16), toll like receptor (TLR2; MCC score = 15), TLR4 (MCC score = 14), IL10 (MCC score = 14), C-X-C motif chemokine ligand 8 (CXCL8; MCC score = 14), and Janus kinase 2 (JAK2; MCC score = 13) (Figure 5(b)).

### 3.5. Molecular Docking of Active Compounds and Pivotal Targets

Molecular docking is a favorable structure-based method to clarify the binding ability of small molecules and interactions between active components and protein targets [45]. Therefore, we utilized molecular docking to further validate the reliability of key targets for Simiao pill treating HUA. In this study, we found 5 overlapping targets (IL1B, IL6, IL10, TLR4, and TNF) from the PPI and GO-KEGG hub gene networks (Figure 6) and 22 active compounds associated with these genes (QED ≥ 0.3) (Table 4).

IL1B, IL6, IL10, TLR4, and TNF were docked with the 22 active compounds, generating 29 decently bound pairs with binding free energy < −5.0 kcal/mol and the formation of hydrogen bonds (Table 5). The top 10 binding pairs (binding free energy ≤ −8.0 kcal/mol) are presented in Figure 7, and other pairs are shown in Figure S1.

### 3.6. HPLC Analysis of the Potential Effective Compounds of Simiao Pill

HPLC analysis was conducted for quality control and identification of the main components of Simiao pill. Herein, chlorogenic acid, magnoflorine, berberine hydrochloride, luteolin, palmitic acid, wogonin, atractylenolide I, osthole, quercetin, rutaecarpine, paeonol, kaempferol, baicalin, vitamin E, and phytosterol were selected for HPLC analysis. Simiao pill is composed of Rhizoma Atractylodis, Cortex Phellodendri, Radix Achyranthis Bidentatae, and Semen Coicis. According to the HIT, TCMSP, and TCMID databases, luteolin, palmitic acid, wogonin, atractylenolide I, and osthole were the active components of Rhizoma Atractylodis; quercetin, rutaecarpine, and paeonol were produced by Cortex Phellodendri; kaempferol, baicalin, and vitamin E were derived from Radix Achyranthis Bidentatae; phytosterol was from Semen Coicis. Chlorogenic acid, magnoflorine, and berberine hydrochloride serve as the signature components for the quality control of Simiao pill. HPLC results showed that luteolin and atractylenolide I were the effective components of Simiao pill compared with those of the mixed standard solution. Furthermore, the proportion of luteolin and atractylenolide I in the sample solution of Simiao pill was 56.2% and 1.39%, respectively (Figure 8).

## 4. Discussion

HUA is a metabolic disease resulting from disordered uric acid metabolism [46]. At present, TCM remains an appealing choice for the treatment of HUA. Some TCM formulas, such as Ermiao Wan [47] and CoTOL [48], have been applied to treat HUA. As a TCM formula, Simiao pill is well-known for its antirheumatic function, which comprises Rhizoma Atractylodis, Cortex Phellodendri, Radix Achyranthis Bidentatae, and Semen Coicis [16]. According to TCM theory, Rhizoma Atractylodis possesses dampness-eliminating and spleen-tonifying functions; Cortex Phellodendri has heat and dampness-eliminating effect; Radix Achyranthis Bidentatae possess liver and kidney-strengthening function; Semen Coicis has spleen-tonifying and diuretic effects [21]. Modern pharmacological research has demonstrated that Simiao pill exerts multiple pharmacological effects, such as anti-inflammatory [22] and uric acid-lowing functions [49]. Otherwise, an *in vivo* study has declared that Simiao pill can alleviate urate underexcretion in HUA mice [50]. These facts prompted us to further explore the curative effects of Simiao pill on HUA. Herein, we employed network pharmacology analysis to find out the mechanisms underlying Simiao pill mitigating HUA. In the current study, we preliminarily identified 264 active compounds of Simiao pill based on ADME screening and 606 relevant target genes. Meanwhile, 303 HUA-related target genes were obtained. Noteworthily, 80 intersection targets related to active compounds of Simiao pill and HUA were acquired for further analysis. Among them, 5 hub genes (IL1B, IL6, IL10, TLR4, and TNF) and 22 relevant active ingredients were identified as underlying molecular interaction mechanisms of Simiao pill treating HUA.

In the PPI network of 80 targets, INS, TNF, IL6, IL1B, VEGFA, LEP, STAT3, CCL2, IL10, and TLR4 were regarded as the top 10 vital targets of Simiao pill treating HUA. Interestingly, some of these core targets were proinflammatory factors, such as TNF, IL6, and IL1B. Evidence has demonstrated that inflammation is significantly implicated in the pathogenesis of HUA [51–53]. Specifically, Nod-like receptor protein 3 (NLRP3) inflammasome is frequently activated during HUA, leading to the secretion of IL1B and other proinflammatory cytokines [52]. Furthermore, an *in vivo* study has indicated that TLR4 inactivation-induced downregulation of TNF, IL6, and IL1B can mitigate the pathological injury of HUA [54]. Additionally, inhibition of the STAT3 signaling pathway can be beneficial to HUA amelioration, as evidenced by relevant studies [55, 56]. These results indicate that Simiao pill may be used to treat HUA owing to its anti-inflammatory function.

At the GO function level, we found that the 80 candidate genes were mainly enriched in BPs, such as response to peptide, regulation of small molecule metabolic process, and positive regulation of cytokine production. Evidence has demonstrated that multiple peptides and proteins are implicated in the onset and progression of HUA [57–60]. A metabolomics analysis-based study has indicated that the pathological mechanisms are associated with the metabolism of various small molecules, such as glycerophospholipid and arachidonic acid [61]. Cytokines have significant implications for the occurrence and development of HUA [62]. For example, an *in vivo* study found downregulation of IL10 (an anti-inflammatory cytokine) in HUA mice, and it showed that upregulation of IL10 inhibited HUA progression [63]. Besides, these targets were closely associated with some MFs, including signaling receptor activator activity and receptor ligand activity. These findings indicate that a wide range of molecules are involved in the pathological mechanisms of HUA, and the regulation of molecular response, production, and metabolism is crucial to HUA progression.

At the KEGG pathway level, our data showed that the mechanisms by which Simiao pill treats UC were primarily related to the AGE-RAGE signaling pathway in diabetic complications and HIF-1 signaling pathway. Accumulating evidence has demonstrated that HUA interacts with type 2 diabetes mellitus [60, 64, 65]. High serum uric acid level can contribute to the development of type 2 diabetes mellitus [64], and glucose metabolism disorder, in turn, can lead to increased serum uric acid [66]. Significantly, the coordination of the advanced glycation end-product (AGE) and its receptor (RAGE) can trigger inflammation [67, 68]. Hypoxia-inducible factor-1 (HIF-1) is one of the core regulators of cellular responses under low-oxygen circumstances [69]. Otherwise, HIF-1*α* is implicated in the regulation of inflammatory factors, such as TNF-*α*, IL1B, and IL-6 [70]. Therefore, the HIF-1 signaling pathway plays a vital part in the inflammatory response. These results indicate that Simiao pill may participate in the treatment of HUA by targeting AGE-RAGE- and HIF-1-related cascade signaling pathways.

Noteworthily, we finally determined 5 core targets according to the PPI and GO-KEGG networks, namely, IL1B, IL6, IL10, TLR4, and TNF. Besides, we found 22 active ingredients of Simiao pill associated with these 5 targets, such as paeonol and wogonin. Crucially, the 5 target proteins exhibited a close affinity with the active compounds, as 29 binding pairs had favorable molecular docking scores of “binding free energy < −5.0 kcal/mol”. Molecular docking results showed that the 12 components kaempferol, luteolin, rutaecarpine, baicalin, quercetin, vitamin E, paeonol, atractylenolide I, osthole, phytosterol, palmitic acid, and wogonin were the pivotal active compounds of Simiao pill in the treatment of HUA. Among these, the active compounds luteolin, quercetin, rutaecarpine, and baicalin displayed strong docking activities with most of the core targets (binding free energy < −7.0 kcal/mol). Also, HPLC analysis was performed to further verify the potential active components of Simiao pill. The results of HPLC analysis showed that luteolin and atractylenolide I were the effective components of Simiao pill. Significantly, luteolin accounted for 56.2%, higher than any other detected compounds in Simiao pill. Combining molecular docking and HPLC analysis, we determined luteolin, rutaecarpine, baicalin, quercetin, and atractylenolide I as the main components of Simiao pill against HUA.

Luteolin belongs to the flavone family, initially found in some fruits and vegetables with potent anti-inflammatory pharmacological function [71]. A previous investigation indicated that luteolin might act on TNF and medicate the HIF-1 pathway implicated in the treatment of HUA [14]. Recent research has indicated that luteolin can effectively reduce the expression of proinflammatory factors IL1B and IL-6 to mitigate TNF-*α*-induced cellular inflammatory injury [72]. Rutaecarpine, an alkaloid extracted from the unripe fruit of E. rutaecarpa, possesses an anti-inflammatory function [73]. Rutaecarpine has been reported to inhibit the expression of IL1B, IL6, and TNF and promote IL10 expression to ameliorate the histopathology damage caused by inflammation [74–76]. Baicalin, a flavonoid compound isolated from radix scutellariae, is characterized by its potent anti-inflammatory effect [77]. Similarly, baicalin can mitigate inflammation by suppressing the expression of IL1B, IL6, and TNF and enhancing IL10 expression [78]. Quercetin is a flavonoid abounding in fruits and vegetables with multiple pharmacological effects, such as antioxidation and anti-inflammation [79]. A recent study has indicated that quercetin may ameliorate HUA by inhibiting TLR4 cascade signaling and downregulating the expression of IL1B, IL6, and TNF [3]. As a eudesmane-type sesquiterpenoid lactone derivative of Rhizoma Atractylodis macrocephalae, atractylenolide I possesses various biological activities, such an-inflammatory and anticancer activities [80]. Evidence has demonstrated the crosstalk between atractylenolide I-induced downregulation of IL1B, IL6, and TNF and TLR4 signaling [81]. Noteworthily, atractylenolide I has been determined as one of the main active components of Rhizoma Atractylodis to treat gouty arthritis via downregulating IL1B, IL6, TNF, and uric acid [82]. Consistent with the previous studies, our data imply that Simiao pill may treat HUA by targeting the release of inflammatory factors and inflammation-related signaling pathways.

However, there are still some limitations in our research. First, we only investigated the potential therapeutic mechanisms of Simiao pill on HUA, without further analyzing the interactions between its active components. Second, the core target genes and pathways were determined at the network pharmacology level and have not been experimentally validated. Third, additional *in vivo* and *in vitro* studies are needed to further verify the efficacy of Simiao pill in treating HUA and its molecular mechanisms. These limitations will be perfected in our subsequent investigations.

## 5. Conclusions

Based on the network pharmacology-molecular docking method, we found that luteolin, quercetin, rutaecarpine, baicalin, and atractylenolide I were the pivotal active ingredients of Simiao pill against HUA, which acted on the key targets, IL1B, IL6, IL10, TLR4, and TNF. This study revealed that Simiao pill could ameliorate HUA mainly by inhibiting inflammation and targeting AGE-RAGE- and HIF-1- associated signaling pathways. There is an essential need for both *in vivo* and *in vitro* experiments to further validate the action mechanisms of the core components of Simiao pill alleviating HUA. Our study provides a direction for the follow-up research into the pharmacological mechanisms of Simiao pill against HUA and offers a reference for the development of novel anti-HUA drugs.

## Figures and Tables

**Figure 1:** Workflow of the network pharmacology and molecular docking-based study.

**Figure 2:** Acquisition of intersection targets related to active components of Simiao pill and HUA using VennDiagram. HUA: hyperuricemia.

**Figure 3:** Construction of PPI network diagram using the STRING database, visualized by ggraph and igraph R packages. Red nodes represent the top 10 hub genes. PPI: protein-protein interaction.

**Figure 4:** GO functional and KEGG pathway enrichment analyses. (a) Fifteen vitally enriched GO functions, including top 5 BP, CC, and MF terms. (b) Top 15 enriched KEGG pathways. *P* value < 0.01. GO: Gene Ontology; KEGG: Kyoto Encyclopedia of Genes and Genomes; BP: biological process; CC: cellular component; MF: molecular function.

**Figure 5:** Identification of 10 hub targets based on GO functional and KEGG pathway enrichment analysis. (a) Construction of the interaction network of candidate targets; top 5 BP, CC, and MF terms of GO enrichment analysis; and top 15 KEGG items. (b) Identification of 10 hub targets corresponding to the GO-KEGG network using the cytoHubba plugin. GO: Gene Ontology; KEGG: Kyoto Encyclopedia of Genes and Genomes.

**Figure 6:** Acquisition of 5 intersection targets from the PPI and GO-KEGG networks of hub targets using VennDiagram. PPI: protein-protein interaction; GO: Gene Ontology; KEGG: Kyoto Encyclopedia of Genes and Genomes.

**Figure 7:** Top 10 well-binding pairs of target protein-active compound through molecular docking.

**Figure 8:** Quality control and main compound validation of Simiao pill through HPLC analysis. (a) Chromatogram of the mixed standard solution (1: chlorogenic acid; 2: magnoflorine; 3: baicalin; 4: berberine hydrochloride; 5: palmitic acid; 6: luteolin; 7: quercetin; 8: kaempferol; 9: paeonol; 10: wogonin; 12: rutaecarpine; 13: osthole; 14: phytosterol; 15: atractylenolide I). (b) Chromatogram of the Simiao pill sample solution (22: luteolin; 27: atractylenolide I). HPLC: high-performance liquid chromatograph.

**Table 1:** Overlapping targets of active components of Simiao pill and hyperuricemia in this study.

ID	Gene name	UniProtKB	ID	Gene name	UniProtKB
1	PPARA	Q07869	41	GAA	P10253
2	HTR2A	P28223	42	G6PC1	P35575
3	P2RX7	Q99572	43	TLR2	O60603
4	FASN	P49327	44	CASP8	Q14790
5	VEGFA	P15692	45	EDN1	P05305
6	ERCC1	P07992	46	SLC22A2	O15244
7	APP	P05067	47	STAT3	P40763
8	TNF	P01375	48	TP53	P04637
9	IL6	P05231	49	EPO	P01588
10	MAPK1	P28482	50	TLR4	O00206
11	NQO1	P15559	51	LPL	P06858
12	MAOA	P21397	52	NOS3	P29474
13	IL1B	P01584	53	IFNG	P01579
14	CYP2E1	P05181	54	CYP11A1	P05108
15	PPARG	P37231	55	INS	P01308
16	ESR1	P03372	56	SLC2A2	P11168
17	SELE	P16581	57	CXCL8	P10145
18	CAT	P04040	58	CRP	P02741
19	MYC	P01106	59	GCG	P01275
20	TGFB1	P01137	60	UCP2	P55851
21	GPT	P24298	61	CYP2C8	P10632
22	IGF1R	P08069	62	PARP1	P09874
23	SOD1	P00441	63	JAK2	O60674
24	SIRT1	Q96EB6	64	CYP2C19	P33261
25	LEP	P41159	65	CD40LG	P29965
26	SERPINE1	P05121	66	ABCG2	Q9UNQ0
27	ADIPOQ	Q15848	67	CCL2	P13500
28	AGT	P01019	68	IL10	P22301
29	POMC	P01189	69	XDH	P47989
30	COL1A1	P02452	70	NLRP3	Q96P20
31	RAPGEF4	Q8WZA2	71	APOE	P02649
32	KHK	P50053	72	ACAT1	P24752
33	GCK	P35557	73	APOB	P04114
34	NGF	P01138	74	COG2	Q14746
35	LCN2	P80188	75	TNFRSF11B	O00300
36	NPPA	P01160	76	ALDH2	P05091
37	NPPB	P16860	77	G6PD	P11413
38	HNF1A	P20823	78	IL6R	P08887
39	HNF4A	P41235	79	IL18	Q14116
40	NFATC1	O95644	80	SLC6A3	Q01959

**Table 2:** Top 5 enriched BP, CC, and MF terms of GO enrichment analysis in this study.

Ontology	ID	Description	*P* value
BP	GO:1901652	Response to peptide	8.27533*E*-26
BP	GO:0062012	Regulation of small molecule metabolic process	1.916*E*-24
BP	GO:0043434	Response to peptide hormone	1.18917*E*-22
BP	GO:0001819	Positive regulation of cytokine production	6.22927*E*-21
BP	GO:0006109	Regulation of carbohydrate metabolic process	5.53126*E*-20
CC	GO:0045121	Membrane raft	8.05101*E*-09
CC	GO:0098857	Membrane microdomain	8.3307*E*-09
CC	GO:0005901	Caveola	4.30163*E*-08
CC	GO:0031983	Vesicle lumen	8.88621*E*-08
CC	GO:0031904	Endosome lumen	2.94786*E*-07
MF	GO:0030546	Signaling receptor activator activity	4.94658*E*-19
MF	GO:0048018	Receptor ligand activity	5.77182*E*-18
MF	GO:0005126	Cytokine receptor binding	3.83607*E*-14
MF	GO:0005125	Cytokine activity	7.90798*E*-14
MF	GO:0005179	Hormone activity	1.25158*E*-10

**Table 3:** Top 15 enriched KEGG pathways of KEGG enrichment analysis in this study.

ID	Description	*P* value
hsa04933	AGE-RAGE signaling pathway in diabetic complications	2.14*E*-17
hsa05417	Lipid and atherosclerosis	2.89*E*-16
hsa05144	Malaria	4.47*E*-16
hsa04066	HIF-1 signaling pathway	1.04*E*-12
hsa05142	Chagas disease	8.03*E*-12
hsa05321	Inflammatory bowel disease	1.53*E*-11
hsa05323	Rheumatoid arthritis	8.42*E*-10
hsa05143	African trypanosomiasis	1.36*E*-09
hsa04932	Nonalcoholic fatty liver disease	1.66*E*-09
hsa05161	Hepatitis B	2.86*E*-09
hsa05145	Toxoplasmosis	6.29*E*-09
hsa04936	Alcoholic liver disease	6.85*E*-09
hsa05146	Amoebiasis	3.30*E*-08
hsa05140	Leishmaniasis	3.58*E*-08
hsa05134	Legionellosis	4.99*E*-08

**Table 4:** Active compounds of Simiao pill related to hub targets.

Pubchem_ID	cpd_name	QED
CID:10228	Osthole	0.61
CID:11092	Paeonol	0.68
CID:12389	Tetradecane	0.37
CID:14985	Vitamin E	0.36
CID:177	Acetaldehyde	0.36
CID:248	Betaine	0.51
CID:440917	Limonene	0.49
CID:5280343	Quercetin	0.43
CID:5280445	Luteolin	0.51
CID:5280863	Kaempferol	0.55
CID:5281515	Beta-caryophyllene	0.5
CID:5281520	Alpha-humulone	0.49
CID:5281703	Wogonin	0.76
CID:5283349	2,4-Decadienal	0.25
CID:5321018	Atractylenolide I	0.47
CID:5997	Phytosterol	0.49
CID:6184	Hexanal	0.39
CID:64982	Baicalin	0.3
CID:65752	Rutaecarpine	0.54
CID:702	Alcohol	0.41
CID:8181	Methyl palmitate	0.3
CID:985	Palmitic acid	0.41

**Table 5:** Results of molecular docking in this study.

Gene	Compound	PubChem ID	Free binding energy (kcal/mol)
IL1B	Kaempferol	CID:5280863	-7.8
	Luteolin	CID:5280445	-7.7
	Quercetin	CID:5280343	-8
	Rutaecarpine	CID:65752	-9.9
	Baicalin	CID:64982	-9.3
	Vitamin E	CID:14985	-6.5
	Paeonol	CID:11092	-5.5

IL6	Atractylenolide I	CID:5321018	-7.3
	Kaempferol	CID:5280863	-7
	Luteolin	CID:5280445	-7.1
	Baicalin	CID:64982	-8.1
	Vitamin E	CID:14985	-6.1
	Osthole	CID:10228	-6
	Phytosterol	CID:5997	-6
	Palmitic acid	CID:985	-5.2

IL10	Quercetin	CID:5280343	-7.3
	Baicalin	CID:64982	-9

TLR4	Wogonin	CID:5281703	-7.8
	Luteolin	CID:5280445	-7.7
	Quercetin	CID:5280343	-8.1
	Rutaecarpine	CID:65752	-8.3

TNF	Atractylenolide I	CID:5321018	-7.7
	Wogonin	CID:5281703	-7.8
	Kaempferol	CID:5280863	-7.8
	Luteolin	CID:5280445	-7.9
	Quercetin	CID:5280343	-8.1
	Rutaecarpine	CID:65752	-8.3
	Baicalin	CID:64982	-8.4
	Vitamin E	CID:14985	-7.1

## Data Availability

The data used to support the findings of this study are available from the corresponding author upon request.

## Supplementary Materials

Supplementary Materials Figure S1: nineteen well-binding pairs of target protein-active compound through molecular docking, apart from the top 10 pairs. Table S1: active components of Simiao pill. Table S2: active components of Simiao pill after ADME screening. ADME: absorption, distribution, metabolism, and excretion. Table S3: targets of active components of Simiao pill. Table S4: targets of hyperuricemia. Table S5: nodes of PPI network. PPI: protein-protein interaction. Table S6: GO enrichment results. GO: Gene Ontology.
